# *DNA Topoisomerase II-α* Regulated by miR-22-5p Promotes Hepatocellular Carcinoma Invasion and Migration through the Hippo Pathway

This article has been retracted.

**DOI:** 10.1155/2022/4277254

**Published:** 2022-10-17

**Authors:** Haichao Zhao, Changzhou Chen, Huangqin Song, Rongyi Qin, Xiaoxiao Wang, Qizu He, Feng Li, Haoliang Zhao, Yanjun Li

**Affiliations:** ^1^Shanxi Bethune Hospital, Shanxi Medical University, Taiyuan 030032, China; ^2^Department of Liver Surgery and Transplantation, Liver Cancer Institute, Zhongshan Hospital, Fudan University, Shanghai 300032, China

## Abstract

*DNA topoisomerases* (*TOPs*) are dysregulated in various types of cancer. However, how *TOP II-alpha* (*TOP2A*) contributes to hepatocellular carcinoma (HCC) progression remains elusive. Cohort analysis revealed that the increased expression of *TOP2A* was associated with poor clinical outcomes and *TOP2A* was significantly upregulated in HCC tissues and cell lines. *In vitro*, *TOP2A* expression level is related to cell invasion and migration, which may be due to the alteration of epithelial-mesenchymal transition by the TOP2A. Moreover, we used verteporfin (a Hippo inhibitor) to test how the Hippo pathway promotes the effect of *TOP2A* on the HCC phenotype and found that *TOP2A* induces tumor progression through the Hippo pathway. Finally, miR-22-5p inhibited tumor progression by sponging *TOP2A*.

## 1. Introduction

Primary liver cancer (PLC) is the sixth most prevalent type of cancer and the fourth leading cause of cancer-related deaths worldwide [1]. Due to the insidious onset and rapid progression of PLC, many patients are diagnosed at an advanced stage [2, 3]. Furthermore, 75% of PLC patients have hepatocellular carcinoma (HCC) [4]. Therefore, identification of cancer-dependent genes that promote HCC progression is essential for HCC treatment.

*DNA topoisomerase II-alpha* (*TOP2A*) encodes DNA topoisomerase, which is the key enzyme for the selective cutting, rearrangement, and reconnection of DNA strands [5]. *TOP2A* is necessary for managing DNA supercoiling and chromosomal separation. It plays important roles in mitosis, including chromosome separation during DNA transcription and replication, chromatin compaction, and torsional stress relief [6]. A previous meta-analysis found that mutation (amplification or deletion) of the *TOP2A* gene leads to shorter survival time of cancer patients [7]. The abnormal expression of TOP2 protein was significantly associated with tumor resistance to adriamycin [8]. The overexpression of *TOP2A* results in accelerated tumor progression and a poor prognosis in lung adenocarcinoma [9]. High TOP2A expression is a favorable prognostic factor in colorectal cancer [10]. Currently, there are no available medications that specifically target TOP2A and its related pathways. Anthracycline medications are the only available empirical drugs, which showed poor efficacy in clinical practice [11].

Dysregulation of the Hippo signaling pathway promotes cancer progression [12, 13]. Moya et al. [14] found that the activity of yes-associated protein (YAP) and transcriptional coactivator with PDZ-binding motif (TAZ) in tumors was linked to the progression of liver tumors. The abnormal activation of the Hippo pathway upregulated androgen receptor (AR) activity in metastatic prostate cancer and reduced the overall survival (OS) of patients [15]. Through enrichment analysis, we identified that TOP2A regulated the cell cycle and DNA replication through the Hippo signaling pathway.

In this study, we aimed to explore the TOP2A tumor-promoting effects and elucidate whether TOP2A regulates the activity of YAP1 in the Hippo signaling pathway by binding to *β*-catenin to exert biological effects. Furthermore, we aimed to explore the mechanisms underlying the high expression of TOP2A and identify the possible targeted drugs.

## 2. Materials and Methods

### 2.1. Data Resource

The mRNA expression and clinical data were obtained from the Cancer Genome Atlas (TCGA) liver cancer dataset (https://www.proteinatlas.org/). We obtained 374 HCC tissue samples and 50 normal liver tissue samples. Fifty nontumor liver tissue samples and 50 HCC tissue samples were obtained from the same patients. Of the 374 participants, 3 had missing data on T stage. Moreover, the data of 110 normal liver tissue samples were obtained from Genotype Tissue Expression (https://xenabrowser.net/hub/). The biological relationship between the two genes was analyzed using Pearson's correlation coefficient (*r*). The moderate or high expression of *TOP2A* coexpressed genes was identified based on the screening criteria (*P* < 0.001, |*r*| > 0.5).

### 2.2. Weighted Gene Coexpression Network Analysis (WGCNA)

The median TOP2A mRNA level was used as an external attribute to categorize the samples into elevated and reduced expression groups, from which the corresponding gene modules could be identified. A gene coexpression network was developed to investigate the modules that were significantly relevant to the sample characteristics. A soft thresholding power of 5 was chosen to generate a weighted network. Except for the gray module, the enlisted genes were grouped into 12 modules. Five of these studies showed high correlation coefficients. These candidate modules were selected for pathway enrichment analysis using the cluster profile package [16].

### 2.3. Patients

This study was approved by the Ethical Review Committee of Shanxi Bethune Hospital (no.: SBQLL-2020-038). Our study included two independent cohorts of 28 patients with HCC at the Shanxi Bethune Hospital (Taiyuan, China). Cohort 1 consisted of 10 randomly selected HCC patients who underwent resection between 2016 and 2019. The paraffin-embedded tissue samples collected from cohort 1 were subjected to immunohistochemistry (IHC). Eighteen patients with HCC in cohort 2 underwent resection between January and December 2020 at the Shanxi Bethune Hospital (Taiyuan, China). The snap-frozen tumor tissues collected from cohort 2 were subjected to quantitative real-time polymerase chain reaction (qRT-PCR) and western blot analysis.

### 2.4. Cell Lines and Cell Transfection

The normal liver cell line L02) and HCC cell lines (MHCC97H, MHCC97L, HCCLM3, SMMC7721, BEL-7404, HepG2 SK-EP-1, and Huh7) were obtained from the Typical Culture Centre Reserve (Shanghai, China). All cells were cultured in Dulbecco's modified Eagle medium (DMEM) supplemented with 10% fetal bovine serum (FBS) (Gibco, Carlsbad, CA, USA), 100 U/ml penicillin, and 100 mg/ml streptomycin (Sigma-Aldrich, St. Louis, MO, USA) in a controlled humidified incubator at 5% CO_2_ and 37°C.

For cell transfection, 0.25 *μ*M small interfering RNA (siRNA; Ribobio, Guangzhou, China) was diluted with 25 *μ*l serum-free Opti-MEM (Gibco, Invitrogen, Carlsbad, CA, USA), gently mixed, and then incubated at 14°C for 5 min. Meanwhile, 25 *μ*l serum-free Opti-MEM was added to 0.5 *μ*l Lipofectamine 2000 (Invitrogen, CA, USA), and the mixture was incubated at 14°C for 5 minutes after being gently mixed. Then, the siRNA and Lipofectamine were incorporated, carefully mixed, and incubated at 14°C for 20 min. Wells were seeded with the siRNA-Lipofectamine mixture containing 50 *μ*l Opti-MEM and gently mixed. After incubation at 37°C for 4–6 hours, fresh DMEM containing 5% FBS without antibiotics was added to the cells after aspirating the medium of the siRNA-Lipofectamine 2000 mixture, and the mixture was incubated for another 24 h. The miRNA mimics were imported from RiboBio (Guangzhou, China).

### 2.5. RNA Extraction and qRT-PCR

TRIzol reagent was used for isolation of total RNA from the tissues and cells (Invitrogen, CA, USA). We used the RT kit M5 Sprint qPCR with gDNA remover (Mei5bio, China) to reverse-transcribe mRNA into cDNA. The first-strand cDNA of miRNA TransScript SuperMix (TransGen Biotech, China) was used for the synthesis of miRNA cDNA. qRT-PCR was performed on a 7500 Fast RT-PCR System (Applied Biosystems, CA, USA) using the SYBR Premix EX Taq II (Takara, Tokyo, Japan). The U6 served as the control for standardizing miRNA, and ATCB was used as the control to standardize mRNA (Table S1).

### 2.6. Western Blot Analysis

Radioimmunoprecipitation assay lysis buffer was used for isolation of proteins from cells (Boster, Wuhan, China), while a bicinchoninic acid kit (Boster, Wuhan, China) was used for determination of protein concentration; the protein samples were heated after being combined with a loading buffer (Boster) at a 5 : 1 ratio. The proteins in the gels were translocated in polyvinylidene difluoride membranes after separation by sodium dodecyl sulfate-polyacrylamide gel electrophoresis. The membrane was incubated with primary antibodies after blocking with 5% nonfit milk powder for 2 h at room temperature (RT). The primary antibodies were used for the analysis after incubating the proteins with the following secondary antibodies: rabbit anti-TOP2A (1 : 2,500; CST, 12286), rabbit anti-E-cadherin (1 : 10,000) (ab40772), rabbit anti-N-cadherin (1 : 10,000) (ab18203), rabbit anti-vimentin (1 : 5,000; Abcam ab92547), rabbit anti-Snail1 (1 : 1,000; Boster, PB0449), rabbit anti-Snail2 (1 : 2,000; Boster, PB9439), rabbit anti-*β*-actin (1 : 10,000; Boster, BM0627), and rabbit anti-GAPDH (1 : 2,000; Boster, A00227-1). The secondary antibodies (1 : 10,000) were purchased from Proteintech, China. The experiments were repeated three times. Finally, the amplified chemiluminescent system was used to visually detect the signal.

### 2.7. Immunohistochemistry

After initial treatment with 4% paraformaldehyde, the tumor tissue was embedded in paraffin and then sliced into 5 *μ*m thick sections. The sections were blocked with 10% goat serum and incubated overnight with anti-TOP2A (1 : 200, 12286, CST) antibody at 4°C. After washing with PBS, the tissue slices were incubated at RT for 1 hour with a secondary antibody that had been conjugated with anti-rabbit or anti-mouse horseradish peroxidase. The paraffin sections were stained with diaminobenzidine and hematoxylin. The IHC slides were observed under a microscope (Nikon, Japan).

### 2.8. Wound Healing Assay

In wound healing studies, cells (5 × 10^4^/500 *μ*l) in the logarithmic growth phase were grown until reach 100% confluence was reached in 24-well plates over a 24-hour course. In the middle of each well, a scratch was made in the HCC cell layer using a 10 *μ*l micropipette tip (denoted as 0 h). To inhibit proliferation, the cells were cultivated in DMEM containing 1% FBS. The HCC cells were gently washed with PBS and cultivated for another 24 h at 37°C in fresh DMEM containing 1% FBS. An inverted light microscope (magnification, 200×; Leica Microsystems, Inc.) was used to photograph the scratched cells. We quantified the extent to which the cells could migrate. We assessed the progress of wound healing and compared the results with the initial measurements. All experiments were independently replicated three times.

### 2.9. Transwell Assay

The invasion ability of HCC cells was evaluated by Transwell assay. Serum-free medium was used for cell starvation for 24 h. HCC cells 2 × 10^4^ cells in 200 *μ*l serum-free media were implanted in the upper chamber (8.0 *μ*m pore size; Corning, Inc.) that was precoated for 8 h with 90 *μ*l Matrigel (BD Biosciences) at 37°C. The lower chamber was then refilled with 600 *μ*l of Roswell Park Memorial Institute 1640 medium (Boster, Wuhan) with 10% FBS and incubated at 37°C for 24 h. Approximately 4% polymethanol (Boster, Wuhan) was used to fix the upper chambers for 30 min before being dyed with 0.1% crystal violet for half an hour at RT. An inverted light microscope was used to photograph the cells that had passed through the membrane and infiltrated into the top chamber. The number of invading or migrating cells was determined by selecting five fields at random.

### 2.10. Dual-Luciferase Reporter Assay

MHCC97L cells were plated in 24-well plates at a density of 1 × 10^5^ cells/well in 0.5 ml. To assess whether miR-22-5p targets TOP2A, 10 ng of wild-type miRNA was transfected into the cells. (TOP2A 3′UTR-WT) or mutant type (TOP2A 3′UTR-Mut) plasmids coexpressing firefly luciferase, 20 pmol of miR-22-5p mimic or NC mimic, and 10 ng of pRL-TK plasmid (Promega, Madison, WI, USA). Lipofectamine RNAi MAX reagent (HANBIO, Wuhan, China) was used to transfect the cells according to the manufacturer's protocol. Using the Dual-Glo luciferase reporter assay system (Promega), the levels of firefly luciferase was compared to that of Renilla luciferase activity, and the F-Luc/R-Luc was determined. Each transfection was performed in triplicate.

### 2.11. Molecular Docking

In this study, Schrödinger (LSA, USA) was used to simulate and dock the screened drugs. The two-dimensional (2D) structure mol2 files of the small molecules were retrieved from DrugBank (https://www.drugbank.com/). The LigPrep module was employed for ligand processing with a pH value of 7.0 ± 2.0. Then, the tautomer status was determined using the Epik program, while the rest of the parameters were used as the default settings of the system. The molecules were optimized using the OPLS2005 force field. The TOP2A number was 1LWZ, according to the keyword search in the Protein Data Bank (PDB, https://www.rcsb.org/). First, Schrödinger's Protein Preparation Wizard module was used for preparatory processing of the protein structure. The system was then optimized using the OPLS3 force field. To produce the ground-state tautomer, the cocrystal ligand pH was adjusted to 7.0 ± 3.0. The Receptor Grid Generation module was used to determine the docking area, while the space position defined the active pocket, which was used as the center of the grid. The ligand-docking module performs ligand docking and sets the conformation and flexibility of the ligand molecule. Finally, various binding modes were scored and sorted based on the molecular energy of docking, and the docking conformation of the molecule was determined based on the lowest docking energy. All small molecules in the small-molecule active ingredient database established above were selected as candidate ligands and docked to the optimized TOP2A protein. Small-molecule active ingredients with high scores were selected. The reported small-molecule active ingredients were selected through literature research to optimize the docking results, narrow the scope of subsequent experimental verification, and improve the pertinence, accuracy, and success rate of small-molecule active component screening.

### 2.12. Statistical Analysis

Data obtained from at least three independent experiments were analyzed using GraphPad Prism 8 (GraphPad Software, Inc., San Diego, CA, USA). The statistical significance between two groups was analyzed using Student's *t*-test. Multiple groups were compared using one-way analysis of variance and Tukey's post hoc test. Means ± standard deviation (SD) were used to display all data. A *P* value of < 0.05 was considered significant.

## 3. Results

### 3.1. High Expression of *TOP2A* as a Predictor of Poor Clinical Outcomes in HCC Patients

*TOP2A* was highly expressed in a variety of tumors (Figure S1), particularly HCC (Figure S2A–C), and the mutation rate in HCC was 76% (Figure 1(a)). Significant differences were observed in the T stage, pathological stage, histological grade, and alpha-fetoprotein (AFP) between the TOP2A^high^ and TOP2A^low^ groups (Table S2). The TOP2A expression levels in T3 and T4 samples were higher than those in T1 and T2 samples (Figure S2D). TOP2A expression was correlated with clinical stage, histological grade, and AFP level (Figure S2E–H). The receiver operating characteristic curve analysis established a good diagnostic value for TOP2A (AUC = 0.951, Figure S2I). The Kaplan-Meier plotter demonstrated that the OS, disease-specific survival, and progression-free interval of patients with high TOP2A expression were reduced (Figure S2J–L). The univariate and multivariate Cox regression analyses revealed that TOP2A expression can be used as an independent predictor of OS (Table S3). Results of the weighted gene coexpression network analysis (WGCNA) revealed that *TOP2A*-related genes were enriched in DNA replication, oocyte meiosis, and the p53 signaling pathway (Figures 1(b)–1(e)). Therefore, TOP2A highly expressed in liver cancer was closely related to high disease grade, late disease stage, and poor prognosis.

### 3.2. Level of *TOP2A* Expression in HCC and Its Relation to the Tumor Volume

IHC analysis confirmed a higher level of *TOP2A* in HCC (Figures 2(a) and 2(b)). RNA and protein were extracted from 18 pairs of HCC tissue samples. Cancer tissues had higher TOP2A mRNA and protein expression levels than the adjacent nontumor tissues (ANT), as shown on qRT-PCR and western blot analysis (Figures 2(c) and 2(d)). The average tumor diameter in the TOP2A^high^ group was higher than that in the TOP2A^low^ group (Figure 2(e)). These results demonstrated that the *TOP2A* expression levels were significantly increased in HCC tissues and were associated with the tumor volume.

### 3.3. Knockdown of TOP2A Suppressing HCC Invasion and Migration In Vitro

To determine the biological functions of TOP2A in HCC cells, we initially detected the expression of *TOP2A* in L02 and 8 HCC cell lines (MHCC97L, MHCC97H, HCCLM3, SMMC7721, BEL-7404, HepG2, SK-HEP-1, and Huh7). The *TOP2A* mRNA and protein expression levels in HCC cell lines were higher than those in L02 cells (Figures 3(a) and 3(b)). MHCC97L and BEL-7404 demonstrated the highest endogenous mRNA and protein expression levels of TOP2A, whereas HepG2 and SK-HEP-1 cell lines demonstrated the lowest TOP2A expression levels (Figures 3(a) and 3(b)). TOP2A knockdown and control MHCC97L and BEL-7404 cell lines were constructed (Figures 3(c) and 3(d)). Results of Transwell and wound healing assays showed that the invasion and migration of HCC cell lines were inhibited by si-*TOP2A* (Figures 3(e) and 3(f)). Silencing of TOP2A increased the E-cadherin expression, accompanied by the downregulation of N-cadherin, vimentin, Snail1, and Snail2 (Figure 3(g)). These results indicate that TOP2A enhances HCC cell invasion and migration via epithelial-mesenchymal transition (EMT).

### 3.4. TOP2A Overexpression Promotes Invasion and Migration of HCC Cells

To further investigate the effects of TOP2A on HCC, we transfected SK-HEP-1 (TOP2A low expression) with the empty vector plasmid (Ctrl group) and the TOP2A recombinant plasmid (TOP2A group) (Figures 4(a) and 4(b)). Results of Transwell assays showed that the TOP2A overexpression increased the invasive ability of SK-HEP-1 cells (Figure 4(c)). Similarly, the recombinant TOP2A plasmid induced the production of SK-HEP-1 cells with stronger migration ability (Figure 4(d)). Western blot analysis results showed that the overexpression of TOP2A decreased the E-cadherin expression and increased the expression of N-cadherin and vimentin, which may have promoted the EMT process by increasing the levels of Snail1 and Snail2 (Figure 4(e)). These results indicated that TOP2A promotes the invasion and migration of HCC cells.

### 3.5. TOP2A Affecting HCC Tumor Progression through Hippo Signaling Pathway

Oncogenes often promote tumor progression by regulating the signaling pathways [12, 13]. Kyoto Encyclopedia of Genes and Genomes (KEGG) enrichment analysis showed that TOP2A was associated to cell cycle, progesterone-mediated oocyte maturation, p53 signaling pathway, and Hippo signaling pathway (Figure 5(a)). Therefore, we speculated that TOP2A exerted tumor-promoting effects through the Hippo pathway. Subsequently, we verified the correlation between TOP2A and key proteins of the Hippo signaling pathway using ENCORI and found that TOP2A was positively correlated with LAST1/2, YAP1, TAZ, and TEAD4 (Figure S3A-E).

Verteporfin (VP), an inhibitor of the Hippo pathway, prevents the binding of YAP and TEAD4 (Figure 5(b)) [16]. Investigations on wound healing revealed that the cell migration ability of MHCC97L and BEL-7404 cells with VP was lower than that of the cells without VP (Figure 5(c)). And VP can inhibit the promigratory effect of TOP2A overexpression (Figure 5(c)). In Transwell experiments, VP inhibited the invasion of HCC cell lines and reversed the TOP2A-mediated promoting effects on HCC cells (Figure 5(d)). Taken together, these results demonstrate that TOP2A promotes HCC development primarily by inactivating the Hippo signaling pathway.

### 3.6. *TOP2A* as a Direct Downstream Target of miR-22-5p

Dysregulation of target gene expression in tumor cells is mainly due to the action of microRNA (miRNA) [17, 18]. Therefore, we explored whether miRNAs affect the HCC growth and metastasis by binding to TOP2A. First, we used miRNA target prediction tools to identify four potential miRNAs (has-miR-139-5p, has-miR-22-5p, has-miR-4683, and has-miR-582-3p) that might bind to TOP2A (Figure 6(a)). TCGA data showed that these candidate miRNAs had low expression in tumor tissues and high expression in ANT (Figure S4A). Patients with elevated levels of miR-139-5p and miR-22-5p had longer OS, while those with higher miR-582-3p levels had shorter OS (Figure S4B). No significant difference was observed in the expression of miR-4683 (Figure S4B). Only hsa-miR-22-5p expression was associated with TOP2A levels (*r* = −0.223, *P* = 4.78*e* − 2; Figure S4C). The expression of the four miRNAs was lower in HCC tissues than in ANT tissues (Figure 6(b)). Results of the qRT-PCR and western blot analysis confirmed that the miR-22-5p expression was significantly associated with reduced TOP2A levels in MHCC97L and BEL-7404 cells (Figures 6(c) and 6(d), Figure S4D). Subcellular localization analysis revealed that miR-22-5p was mainly expressed in the cytoplasm (Figure 6(e)). miR-22-5p mimics reduced the migration and invasion abilities of MHCC97L and Bel-7404 cells (Figures 6(f) and 6(g)). Overexpression of miR-22-5p in MHCC97L and BEL-7404 cells reduced the levels of E-cadherin, YAP1, p-YAP1, and TEAD4 (Figure 6(h)). The overexpression of miR-22-5p reduced the luciferase activity in the wild-type LUC-TOP2A reporter gene, while it had had no significant effect on the mutant LUC-TOP2A type (Figure 6(i)). Together, these findings indicate that TOP2A is a direct target of miR-22-5p in HCC cells, and the overexpression of miR-22-5p suppresses the invasion and migration of HCC cells.

### 3.7. TOP2A Overexpression Reversing the Effect of miR-22-5p

miR-22-5p inhibited the expression of TOP2A by binding to the 3′UTR of TOP2A mRNA. A decrease in the mRNA and protein levels of TOP2A was induced by miR-22-5p mimics. TOP2A overexpression reversed these effects (Figures 7(a) and 7(b)). The results of wound healing experiments showed that mi-22-5p inhibited the migration ability of MHCC97L and BEL-7404 cells, but this inhibition was reversed by the overexpression of TOP2A (Figure 7(c)). Likewise, TOP2A overexpression reversed the invasion-suppressive effect of miR-22-5p on MHCC97L and BEL-7404 cells (Figure 7(d)). Collectively, these results indicated that miR-22-5p downregulated the expression of TOP2A, thereby exerting a tumor suppressor effect. TOP2A overexpression reversed the effect of miR-22-5p.

### 3.8. Refametinib and Dabrafenib as Effective Drugs Targeting TOP2A

We explored the TOP2A interactions using the data obtained from the DrugBank for drug-protein effect analysis (Figure S5). Molecular docking showed that two TOP2A inhibitors, teniposide and etoposide, did not show high binding power, whereas refametinib (high extra precision) and dabrafenib (high standard precision) showed stronger binding power and effect on TOP2A (Table 1, Figure 8). These results demonstrated that refametinib and dabrafenib can be used as potential targeted drugs for TOP2A.

## 4. Discussion

Inactivation of the Hippo signaling pathway is pivotal for cancer onset and progression. In this study, TOP2A was identified as an oncogenic gene that is highly expressed in HCC by inhibiting the Hippo signaling pathway. The upregulation of TOP2A, which promoted EMT, is responsible for the promotion of HCC cell invasion and migration. Mechanistically, TOP2A altered the invasiveness and migration of HCC cells through the Hippo signaling pathway. Moreover, the lack of miR-22-5p led to an abnormal increase in the levels of TOP2A expression in HCC cells. Taken together, our study unravels the hitherto unappreciated role of TOP2A in the Hippo signaling pathway.

Chromosomal instability (CIN) is a major feature of cancer cells and is associated with DNA unwinding and mutations and epigenetic modifications of repair genes (topoisomerase family genes) [6]. In the TCGA LIHC cohort, the mutation rate of TOP2 was much higher than that of TOP1 and TOP3. TOP2 is expressed in most eukaryotic organisms and has two isoforms, namely, TOP2A and TOP2B [19]. TOP2A is mainly active during DNA replication and mitosis [20], while TOP2B participates in the transcriptional regulation of gene expression [21]. In various types of tumors, including HCC, TOP2A shows huge expression differences. TOP2A expression is correlated with tumor resistance [22–24]. In 2019, Peng et al. [25] found that a small group of malignant cells from pancreatic ductal adenocarcinoma sample expressed *MKI67*, *TOP2A*, and *CCNB1*, and these cells showed a high degree of malignancy to promote tumor progression. TOP2A was dysregulated in other tumor types [26]. However, there are few studies on TOP2A in the field of liver cancer, all of which are bioinformatics research [27, 28]. In this study, we investigated the cancer-promoting effects of TOP2A on HCC. The overexpression of TOP2A stimulated the invasion and migration of HCC cells and accelerated the liver cancer progression.

In the WGCNA analysis, TOP2A was mainly associated with DNA replication. Consistent with the findings of this analysis, we observed that TOP2A overexpression in HCC cells upregulated the levels of Snail1 and Snail2 and increased those of N-cadherin and vimentin. TOP2A promotes EMT in HCC cells to increase their invasion and migration capabilities. Wang et al. [29] confirmed that TOP2A in cervical cancer promotes EMT in tumor cells through the PI3K/AKT signaling pathway, which leads to tumor metastasis. Collectively, these results illustrated that TOP2A enhance the motility of HCC cells through EMT.

KEGG enrichment and GSEA analysis were conducted to investigate the mechanism by which TOP2A promotes the HCC progression. Results showed that TOP2A and its related genes were enriched in the Hippo signaling pathway. The Hippo signaling pathway controls organ growth by suppressing cell growth and stimulating apoptosis. The dysregulation of the pathway often leads to uncontrolled cell division in various cancer types [30]. The Hippo pathway is crucial for the initiation of liver cancer [31]. Through the use of verteporfin (VP), we were able to perform cell experiments and further validate the connection between the TOP2A pathway and the Hippo pathway. VP is a photosensitizer of photodynamic therapy (PDT) and was identified as an inhibitor of the combination of YAP1 and TEAD4 [32]. We found that VP inhibits HCC cell invasion and migration induced by TOP2A overexpression. TOP2A promotes tumor progression through the Hippo pathway. Weiler et al. [33] found that activating YAP can induce CIN. Conversely, disrupting the interaction between YAP and TEAD4, the transcriptional coactivators of the Hippo signaling pathway, reduces the expression of CIN genes (including TOP2A). TOP2A affects the mobility of HCC cells through the Hippo signaling pathway.

Dysregulation of miRNAs occurs in most tumor cells [34]. miRNA and mRNA often form a complex ceRNA network to regulate the expression of oncogenes in tumors [35]. The level of miR-22-5p was relatively low in HCC tissues and reduced the TOP2A expression by binding to the mRNA 3′UTR region. Consistent with these reports, miR-22-5p mimics reduced the HCC cell proliferation, migration, and invasion, in addition to inducing apoptosis, which was rescued by the overexpression of TOP2A. Han et al. [36] found that MIR22HG upregulated the expression of miR-22-3p and miR-22-5p in the cytoplasm and affected the progression of gliomas via the Wnt/*β*-catenin signaling pathway. In summary, the reduction of miR-22-5p level in HCC cells may be the reason for the high TOP2A expression.

With the advancement of molecular structure determination technology, the use of molecular docking to identify specific binding drugs for target proteins has improved the efficiency of clinical translation [37]. To identify the application of TOP2A as a therapeutic target in HCC, we employ network pharmacology to identify drugs that can affect the TOP2A and predict the effective binding site. Anthracyclines can be applied to TOP2A, but their efficacy is mild [11]. We screened nine drugs that act on TOP2A to evaluate the receptor-ligand binding conformation and affinity through molecular docking. Results showed that dabrafenib and refametinib have higher TOP2A affinities compared with traditional anthracyclines. Therefore, we assessed the clinical benefits of dabrafenib and refametinib.

However, our study has some limitations. TOP2A plays a regulatory role in HCC via the Hippo signaling pathway, but its specific details have not been clearly explored. The key point of Hippo signaling pathway in which TOP2A acts through needs to be explored further. Furthermore, in vivo experiments should be conducted to elucidate this specific mechanism.

## 5. Conclusion

In summary, we have identified TOP2A as a crucial promoter of HCC progression. TOP2A affects HCC cell EMT through the Hippo signaling pathway to promote HCC invasion and migration. High TOP2A expression levels were associated with a reduction in the expression of miR-22-5p. Therefore, TOP2A may be a biomarker for predicting the prognosis and a target for HCC therapy.

## Figures and Tables

**Figure 1:** Genomic analysis of TOPs in HCC and WGCNA predicted biological pathways associated with TOP2A. On the basis of GSE121248's expression profile, WGCNA was used to cluster genes that were highly connected with high TOP2A group and low TOP2A group. (a) OncoPrint visual summary of change on a query of TOPs and the high mutation rate of TOPs in HCC patients were detected (cBioPortal). (b) The cluster dendrogram of coexpression network modules. (c) The gene clusters obtained by the WGCNA method. (d) Significantly enriched biological process of the co-expressed genes in yellow module. (e) A network diagram showing significantly enriched biological process of the coexpressed genes in the yellow module using Metascape.

**Figure 2:** *TOP2A* was highly expressed in HCC tissues and correlated to the tumor volume. (a) Representative images of *TOP2A* expression in HCC tissues and ANT. Scales represent 50 micron. (b) Histogram of IHC image optical density quantification. (c) Connection diagram of *TOP2A* mRNA expression in 18 paired tissues. (d) *TOP2A* protein expression level in 18 paired HCC tumor tissues (C) and their adjacent normal tissues (N). Histogram of western blot analysis (right). (e) Histogram of the largest tumor diameter in the TOP2A^high^ and TOP2A^low^ groups. Data are presented as mean ± SEM; ^∗∗∗^*P* < 0.001, ^∗∗^*P* < 0.01, and ^∗^*P* < 0.05.

**Figure 3:** *TOP2A* knockdown inhibited the invasion and migration of HCC cell lines. (a) The mRNA level of TOP2A in normal liver cell lines and HCC cell lines was determined by RT-qPCR. (b) The protein expression of TOP2A in normal liver cell lines and HCC cell lines was determined by western blot analysis. (c) The TOP2A expression level in MHCC97L and BEL-7404 cells transfected with siRNAs targeting TOP2A was assessed by RT-qPCR. (d) The TOP2A expression level in MHCC97L and BEL-7404 cells transfected with siRNAs targeting TOP2A was determined by western blot analysis. (e) Transwell invasion assay of HCC cells transfected with si-Ctrl or si-TOP2A. The bar graphs show the number of migrating and invasive cells after 24 h. (f) Representative images of wound healing assays after scratch wounding of the cells described. (g) Western blot analysis was performed to detect the expression of EMT-related protein in HCC cells transfected with si-Ctrl or si-TOP2A. Data are shown as mean ± SEM; ^∗∗∗^*P* < 0.001, ^∗∗^*P* < 0.01, and ^∗^*P* < 0.05.

**Figure 4:** *TOP2A* overexpression promotes HCC *invasion and migration in vitro*. (a) TOP2A expression in SK-HEP-1 cells transfected with TOP2A was determined by RT-qPCR. (b) Western blot analysis of indicated HCC cells (SK-HEP-1) transfected with TOP2A-vector (Ctrl group) or TOP2A (TOP2A group). (c) Transwell invasion assay of HCC cells transfected with Ctrl or TOP2A. The bar graphs show the number of migrating and invasive cells after 24 h. (d) Representative images of wound healing assays after scratch wounding of the cells described. (e) Western blot analysis was performed to detect the epithelial mesenchymal protein expression in HCC cells transfected with Ctrl or TOP2A. Data are shown as mean ± SEM; ^∗∗∗^*P* < 0.001, ^∗∗^*P* < 0.01, and ^∗^*P* < 0.05.

**Figure 5:** *TOP2A* affects HCC tumor progression through the Hippo signaling pathway. (a) KEGG enrichment analysis of TOP2A related pathways. (b) VP inhibits the Hippo signaling pathway. (c) Wound healing assays of HCC cells treated with Ctrl+DMSO, Ctrl+VP 1 *μ*g/ml, Ctrl+VP 2 *μ*g/ml, TOP2A+DMSO, TOP2A+VP 1 *μ*g/ml, and TOP2A+VP 2 *μ*g/ml. (d) Transwell invasion assay of HCC cells treated with Ctrl+DMSO, Ctrl+VP 1 *μ*g/ml, Ctrl+VP 2 *μ*g/ml, TOP2A+DMSO, TOP2A+VP 1 *μ*g/ml, and TOP2A+VP 2 *μ*g/ml. The bar graphs show the number of migrating and invasive cells after 24 h. Data are shown as mean ± SEM; ^∗∗∗^*P* < 0.001, ^∗∗^*P* < 0.01, and ^∗^*P* < 0.05.

**Figure 6:** miR-22-5p inhibits the cancer-promoting effect of TOP2A. (a) Venn diagram shows the miRNAs predicted by the database that can interact with TOP2A mRNA. (b) qRT-PCR revealed the miRNA expression in liver cancer tissues and ADT. (c) qRT-PCR showed that the expression level of TOP2A mRNA in the HCC cell line (MHCC97L) transfected with miRNAs. (d) Western blot analysis demonstrated the TOP2A protein expression in the HCC cell line (MHCC97L and BEL-7404) transfected with miRNAs (e) RNA levels of miR-22-5p, GAPDH, and U6 in the nuclear and cytoplasmic fractions of MHCC97L cells. (f) Wound healing assays of HCC cells (MHCC97L and BEL-7404) transfected with miR-Ctrl or miR-22-5p mimics. (g) Transwell invasion assay of HCC cells (MHCC97L and BEL-7404) transfected with miR-Ctrl or miR-22-5p mimics. The bar graphs show the number of migrating and invasive cells after 24 h. (h) Western blotting was utilized for detection E-cad and Hippo pathway-associated protein expression in HCC cells (MHCC97L and BEL-7404) transfected with miR-Ctrl or miR-22-5p mimics. (i) Dual-luciferase reporter assay to detect the activity of LUC-TOP2A-wt or LUC-TOP2A-mutant in MHCC97L cells after overexpression of miR-22-5p. The predicted binding site of miR-22-5p in TOP2A. The mut sequence contains a 7-base mutation in the miR-22-5p target seed region. The wild-type and a mutated type of binding site between miR-22-5p and TOP2A.Data are shown as mean ± SEM; ^∗∗∗^*P* < 0.001, ^∗∗^*P* < 0.01, and ^∗^*P* < 0.05.

**Figure 7:** *TOP2A* overexpression reverse the effect of miR-22-5p. (a, b) qRT-PCR and western blot analysis exposed the TOP2A mRNA and protein level of HCC cell lines (MHCC97L and BEL-7404) transfected with miR-Ctrl+vector, miR-22-5p mimics+vector, or miR-22-5p mimics+TOP2A. (c) Wound healing assays of HCC cells treated with miR-Ctrl+vector, miR-22-5p+vector, and miR-22-5p+TOP2A. (d) Transwell invasion assay of HCC cells treated with miR-Ctrl+vector, miR-22-5p+vector, and miR-22-5p+TOP2A. The bar graphs show the number of migrating and invasive cells after 24 h. Data are shown as mean ± SEM; ^∗∗∗^*P* < 0.001, ^∗∗^*P* < 0.01, and ^∗^*P* < 0.05.

**Figure 8:** Virtual screening of TOP2A protein inhibitors based on molecular docking. (a) TOPA protein 3D structure. (b) Structure-based TOP2A-drug reaction prediction.

**Table 1:** Information on the nine prospective drugs with significant scores for hepatocellular carcinoma treatment.

Drug name	PubChem CID	Molecular formula	Classification	Docking score	SP^a^	XP^b^
Trametinib	11707110	C_26_H_23_FIN_5_O_4_	Protein kinase inhibitor Antineoplastic agents Immunomodulating agent	-6.885	-6.885	-4.976
Selumetinib	10127622	C_17_H_15_BrClFN_4_O_3_	Tyrosine kinase inhibitors	-6.164	-6.172	-6.844
Refametinib (RDEA119)	44182295	C_19_H_20_F_3_IN_2_O_5_S	Inhibitor of mitogen-activated ERK kinase	-5.403	-5.405	-7.441
PD-0325901	9826528	C_16_H_14_F_3_IN_2_O_4_	ERK MAPK signaling	-6.213	-6.213	-7.227
Dabrafenib	44462760	C_23_H_20_F_3_N_5_O_2_S_2_	Reversible ATP-competitive kinase inhibitor	-4.725	-7.726	-6.128
Navitoclax	24978538	C_47_H_55_ClF_3_N_5_O_6_S_3_	Bcl-2 antagonist	-7.429	-7.588	-5.757
Teniposide	452548	C_32_H_32_O_13_S	Topoisomerase II inhibitors Immunomodulating agents	-4.725	-4.726	-4.803
Etoposide	36462	C_29_H_32_O_13_	Topoisomerase II inhibitors Antineoplastic agents	-4.994	-4.994	-4.078
Neopeltolide	16115403	C_31_H_46_N2O_9_	Inhibitor of mitochondrial ATP synthesis coupled proton transport	-5.752	-5.752	-5.216

^a^SP: standard precision; ^b^XP: extraprecision.

## Data Availability

On reasonable request, the corresponding authors provided access to all data collected and/or analyzed during this investigation.

## Abbreviations

PLC: Primary liver cancer
HCC: Hepatocellular carcinoma
TOP2A: DNA topoisomerases II-alpha
ANT: Adjacent nontumor tissue
CIN: Chromosomal instability
miRNA: MicroRNA
OS: Overall survival
qRT-PCR: Quantitative real-time polymerase chain reaction
EMT: Epithelial-mesenchymal transition
AFP: Alpha-fetoprotein
SCID mice: Severe combined immune deficient mice.

## Supplementary Materials

Supplementary Materials Table S1: fluorescent primer sequences. Table S2: baseline data table based on TOP2A expression from TCGA. Table S3: single/multiple logistic regression analysis of factors associated with TOP2A. Figure S1: the expression of *TOP*s in 33 kinds of tumors. TOPs are unregulated in most tumors, and TOP2A is present huge expression difference in cancerous and non-cancerous tissues in a variety of tumors. (A) Pan-cancer expression of TOP1. (B) Pan-cancer expression of TOP2A. (C) Pan-cancer expression of TOP2B. (D) Pan-cancer expression of TOP3A. (E) Pan-cancer expression of TOP3B. Figure S2: *TOP2A* expression between cancer and normal tissues in HCC. (A) Violin chart showed the expression of T*OP2A* mRNA in primary HCC tissues and normal tissues (TCGA). (B) Connection diagram showed the expression of *TOP2A* mRNA in 50 paired samples. (C) Box plot showed the expression of *TOP2A* mRNA in primary HCC tissues and normal tissues (TCGA+GTEx). (D) Box plot showed the association between *TOP2A* expression and T stage. (E) Box plot showed the association between TOP2A expression and pathologic stage. (F) Box plot showed the association between TOP2A expression and histologic grade. (G) Box plot showed the association between TOP2A expression and AFP. (H) Box plot showed the association between TOP2A expression and tumor status. (I) Receiver operating characteristic (ROC) curves to test the value of TOP2A to identify HCC tissues. (J) Kaplan-Meier survival curves showed Overall survival comparing the high and low expression of TOP2A in HCC patients. (K) Kaplan-Meier survival curves showed disease-specific survival comparing the high and low expression of TOP2A in HCC patients. (L) Kaplan-Meier survival curves showed progression-free interval comparing the high and low expressions of TOP2A in HCC patients. Data are shown as mean ± SEM; ^∗∗∗^*P* < 0.001, ^∗∗^*P* < 0.01, and ^∗^*P* < 0.05. Figure S3: correlation of key proteins in TOP2A and Hippo signaling pathway (ENCORI). (A) Correlation of TOP2A and LAST1 expression in LIHC. (B) Correlation of TOP2A and LAST2 expression in LIHC. (C) Correlation of TOP2A and YAP1 expression in LIHC. (D) Correlation of TOP2A and TAZ expression in LIHC. (E) Correlation of TOP2A and TEAD4 expression in LIHC. Figure S4: correlation analysis of miRNAs (has-miR-139-5p, has-miR-22-5p, has-miR-4683, and has-miR-582-3p). (A) Box plot showed the expression of miRNAs (has-miR-139-5p, has-miR-22-5p, has-miR-4683, and has-miR-582-3p) in primary HCC tissues and normal tissues of LIHC (TCGA). (B) Kaplan-Meier survival curves showed overall survival comparing the high and low expression of miRNAs (has-miR-139-5p, has-miR-22-5p, has-miR-4683, and has-miR-582-3p) in HCC patients. (C) Correlation of TOP2A and miRNAs (has-miR-139-5p, has-miR-22-5p, has-miR-4683, and has-miR-582-3p) expression in 374 LIHC samples (ENCORI). (D) qRT-PCR showed that the expression level of TOP2A mRNA was in the HCC cell line (7404) transfected with miRNAs. Data are shown as mean ± SEM; ^∗∗∗^*P* < 0.001, ^∗∗^*P* < 0.01, and ^∗^*P* < 0.05. Figure S5: 2D images of drugs that can work with TOP2A (DrugBank).
